The article "Specific blockade of Rictor-mTOR association inhibits mTORC2 activity and is cytotoxic in glioblastoma" was retracted in 2023. Reasons: an official misconduct investigation; misconduct by an author; errors in the images; duplicated images.

# Specific blockade of Rictor-mTOR association inhibits mTORC2 activity and is cytotoxic in glioblastoma

**DOI:** 10.1371/journal.pone.0176599

**Published:** 2017-04-28

**Authors:** Angelica Benavides-Serrato, Jihye Lee, Brent Holmes, Kenna A. Landon, Tariq Bashir, Michael E. Jung, Alan Lichtenstein, Joseph Gera

**Affiliations:** 1 Department of Medicine, David Geffen School of Medicine, University of California-Los Angeles, Los Angeles, California, United States of America; 2 Department of Research & Development, Greater Los Angeles Veterans Affairs Healthcare System, Los Angeles, California, United States of America; 3 Department of Chemistry and Biochemistry, University of California-Los Angeles, Los Angeles, California, United States of America; 4 Jonnson Comprehensive Cancer Center, University of California-Los Angeles, Los Angeles, California, United States of America; 5 Molecular Biology Institute, University of California-Los Angeles, Los Angeles, California, United States of America; Emory University, UNITED STATES

## Abstract

A small molecule which specifically blocks the interaction of Rictor and mTOR was identified utilizing a high-throughput yeast two-hybrid screen and evaluated as a potential inhibitor of mTORC2 activity in glioblastoma multiforme (GBM). *In vitro*, CID613034 inhibited mTORC2 kinase activity at submicromolar concentrations and in cellular assays specifically inhibited phosphorylation of mTORC2 substrates, including AKT (Ser-473), NDRG1 (Thr-346) and PKC**α** (Ser-657), while having no appreciable effects on the phosphorylation status of the mTORC1 substrate S6K (Thr-389) or mTORC1-dependent negative feedback loops. CID613034 demonstrated significant inhibitory effects on cell growth, motility and invasiveness in GBM cell lines and sensitivity correlated with relative Rictor or SIN1 expression. Structure-activity relationship analyses afforded an inhibitor, JR-AB2-011, with improved anti-GBM properties and blocked mTORC2 signaling and Rictor association with mTOR at lower effective concentrations. In GBM xenograft studies, JR-AB2-011 demonstrated significant anti-tumor properties. These data support mTORC2 as a viable therapeutic target in GBM and suggest that targeting protein-protein interactions critical for mTORC2 function is an effective strategy to achieve therapeutic responses.

## Introduction

GBM are highly malignant and invasive tumors, properties which prevent total surgical resection, and render these neoplasms refractory to chemotherapeutic interventions [1]. Prognosis for patients is very poor and most succumb to the disease within a year [2]. Patients that do survive typically develope significant long-term toxicities as a result of high-dose chemotherapies ultimately leading to drug resistance [3]. Thus, the development of novel therapeutic options based on the biology of these heterogeneous tumors is necessary while circumventing resistance mechanisms.

The mechanistic target of rapamycin (mTOR) kinase is the major mediator of phosphatidylinositol 3-kinase (PI-3K) signaling and is an important target for molecular therapeutics in GBM [4, 5]. mTOR is a common element in two separate multicomponent kinase complexes [6, 7]. The mTOR-mLST8-Raptor complex (mTORC1) integrates signals regulating cell size and growth whereas the mTOR-mLST8-mSIN1-Rictor complex (mTORC2) regulates cell cycle-dependent cytoskeleton assembly in addition to growth [8]. mTORC2 has emerged as a promising target in GBM, as recent data indicate that mTORC2 activity is essential for the transformation and invasive characteristics of these tumors, yet in many normal cells mTORC2 activity appears nonessential [9–11].

Essential to the successful targeting of mTORC2 is an understanding of the mechanisms of its dysregulation. Constitutive activation of upstream signaling pathways contribute to mTORC2 activation, via growth factors, PI-3K and TSC1-TSC2 activation as has been reported [9]. Recent data demonstrates that association with the ribosome directly can activate mTORC2 [12]. Another mechanism by which cells may regulate mTORC2 activity is by governing the expression levels of essential regulatory subunits. It has been demonstrated that in gliomas increased Rictor expression can be correlated with increased phospho-S^473^-AKT levels [13, 14] and this has now been described in a variety of cancer cell types [15–17]. Moreover, overexpressing Rictor enhances oncogenic traits of tumor cells [14] and genetically engineered mouse model (GEMM) studies demonstrate that it is indeed a *bone fide* oncoprotein [18]. It is frustrating that inhibiting components of the EGFR/PI-3K/AKT/mTORC signaling axis in GBM has proved to be cytostatic rather then inducing cell death or apoptosis, even though AKT and mTOR have clearly established anti-apoptotic roles [3]. More likely then, alternative survival pathways may become activated allowing cells to evade pro-apoptotic signals mediated by EGFR/PI-3K/AKT/mTORC blockade.

The discovery that mTORC2 directly activates AKT led to hypotheses that mTORC2-specific inhibitors may also be valuable anti-cancer drugs [9]. Such a compound, in addition to blocking AKT phosphorylation, would also have the advantage of not disrupting the mTORC1-dependent negative feedback loops, which have now been demonstrated to be a major mode of drug resistance to mTORC1 inhibitors [19, 20]. ATP-competitive inhibitors of mTORC1 and mTORC2 have been developed with the promise that simultaneous inhibition of both mTOR nucleated complexes would be more effective then mTORC1-specific inhibitors, yet these compounds may suffer from toxicity issues as well as continuing problems related to disruption of mTORC1 feedback loops at therapeutic concentrations [9]. Additionally, inhibition of mTORC1 also activates autophagy which may promote glioma cell survival [21, 22].

In this report we describe the identification and characterization of a novel small molecule inhibitor of mTORC2. The inhibitor specifically blocks the interaction of the regulatory subunit Rictor with mTOR and blunts mTORC2 signaling while mTORC1 signaling is unaffected. We show that the inhibitor displays strong anti-GBM effects *in vitro*, blocking growth, motility and invasive characteristics of GBM cell lines. Sensitivity to the inhibitor correlated with elevated Rictor or mSIN1 expression. Structure-activity relationship (SAR) studies led to the identification of an improved mTORC2 inhibitor (JR-AB2-011) and further mechanistic investigations suggested that these compounds bind Rictor and inhibit association with mTOR. Finally, we demonstrate that the JR-AB2-011 inhibitor markedly reduces GBM xenograft growth and blocks mTORC2 signaling in these tumors.

## Materials and methods

### Cell lines, constructs and transfections

The SF763 line was obtained from the UCSF Neurosurgery Tissue Bank and all other lines were from ATCC (Manassas, VA). Normal mature human neurons were obtained from ScienCell (Carlsbad, CA). Wild-type and SIN1-null MEFs were generously provided by Dr. Bing Su (Yale University). Lines were obtained from 2001–2012 and routinely tested to confirm the absence of mycoplasma. Cell authentication by ATCC is done by STR profiling. The myc-Rictor (corrected) and Deptor constructs were gifts from Dr. David Sabatini (Whitehead Institute/MIT) and the Flag-mTOR and mSIN1-HA constructs were gifts from Dr. Jie Chen (University of Illinois). DNA transfections were performed using Effectene transfection reagent according to the manufacturer (Qiagen).

### Recombinant proteins, antibodies, reagents and CID613034 SAR analog preparation

Proteins were expressed and purified from HEK293 cells using anti-myc, anti-HA or anti-Flag Sepharose column chromatography as previously described [23]. Recombinant Raptor was from Abcam (Cambridge, MA) and recombinant mLST8 was obtained from Abnova (Walnut, CA). All antibodies are described in supplemental materials (S1 File). Antimycin A was from Sigma and rapamycin was obtained from LC Laboratories (Woburn, MA). CID613034 (JR-AB2-000) was obtained from the Developmental Therapeutics Program repository at the NCI. Additionally, large-scale amounts of analog JR-AB2-011 (ID# STK377726) was obtained from Vitas-M Ltd., (Champaign, IL). The synthetic procedures for the SAR analogs are described in detail in the supplemental materials (S1 File).

### High-throughput yeast-two-hybrid screening

The yeast two-hybrid strain AH109 was modified to maximize the penetration of small molecules via disruption of *PDR1* and *PDR3* (positive regulators of ABC transporters, which when overexpressed lead to pleiotropic drug resistance) [24]. Simultaneously, the hexose transporters *HXT11* and *HXT9*, which when overexpressed enhances the sensitivity of yeast to small molecules [25], were placed under control of the copper-inducible *CUP1* promoter. This strain was then transformed with constructs containing the human full-length Rictor fused to the GAL4 DNA-binding domain (DBD) and mTOR fused to the GAL4 activation domain (AD). Interaction of Rictor and mTOR reconstituted a functional transcription factor capable of inducing *GAL4*-upstream activating sequence containing reporters and allowed for growth on selective media. Yeast were subsequently interrogated against a >145,000 diversity oriented small molecule library (NCI, Developmental Therapeutics Program) by robotic-aided pinning of compounds onto a lawn of cells. Compounds, which blocked yeast growth, resulted in halo formation and identification of candidate Rictor-mTOR inhibitors. As a counterscreen, we engineered yeast that were dependent on the interaction of the SV40 large T antigen and p53 for growth on selective media and compounds which blocked growth of both strains of yeast were considered nonspecific. In three experiments, the Z' values were between 0.78 and 0.86, consistent with high robustness of the screen.

### Protein expression, co-immunoprecipitation and *in vitro* kinase analyses

Western blot analyses were performed as previously described [14]. Briefly, cells were lysed in RIPA (lysis) buffer containing protease inhibitor cocktail and phosSTOP phosphatase inhibitor cocktail (Roche) and extracts resolved by SDS-PAGE. Proteins were transferred to PVDF membranes and incubated with the indicated antibodies. Antigen-antibody complexes were detected using appropriate horseradish peroxidase-conjugated secondary antibodies (GE Healthcare) and enhanced chemiluminescence (Amersham ECL Prime). Co-immunoprecipitations were performed as previously described [26]. mTORC2 *in vitro* kinase assays were performed as described utilizing GST-tagged AKT as a substrate [14].

### Surface plasmon resonance (SPR) and mTOR-flag binding assays

SPR experiments were carried out on a Biacore 2000 optical biosensor (BioCore AB, Piscataway NJ) using immobilized recombinant Rictor, mSIN1 or mTOR as described [27]. Binding was observed as the change in response units (RU) as analyte was injected at a flow rate of 10 μl/min at 25°C. For SPR competitive solution binding experiments, on an mTOR immobilized CM5 chip, pre-incubated Rictor, Raptor, mLST8 or Deptor with inhibitor (30 min) reaction mixtures were injected over the surfaces of the chip. Response units were measured in the dissociation phase and specific binding was calculated by subtracting the control surface signal from the surfaces with immobilized mTOR. For mTOR-Flag binding assays, purified myc-Rictor was pre-treated with increasing concentrations of JR-AB2-000 or JR-AB2-011 for 1h at 4°C and subsequently added to mTOR-Flag beads and incubated overnight at 4°C. Incubated beads were washed five times and immunoblotted using an anti-myc or anti-Flag antibody as indicated.

### Cell proliferation, cell-cycle distribution and TUNEL assays

Cells were plated into 96-well plates and after culturing for various time points, cell numbers were measured by 2,3-bis[2-methoxy-4-nitro-5-sulfophenyl]-2*H*-tetrazolium-5-carboxanilide inner salt (XTT) assay (Roche) as described by the manufacturer. Viability of human neurons was assessed by trypan blue- exclusion. Cell-cycle analysis was done by propidium iodide staining of cells and flow cytometry as previously described [28]. Cells were stained using a FITC-conjugated annexin V (Annexin V-FITC Early Apoptosis Detection kit, Cell Signaling) to monitor apoptosis. Immunohistochemical staining of tumor sections for Ki-67 was performed as previously described [18]. TUNEL staining of tumor sections was performed using the TACSXL DAB *In Situ* Apoptosis Detection kit (Trevigen) according to the manufacturer’s instructions [28].

### Xenograft studies

All animal experiments were performed under an approved Institutional Animal Care and Use Committee protocol and conformed to the guidelines established by the Association for the Assessment and Accreditation of Laboratory Animal Care. Xenografts of LN229 cells were performed in female C.B.-17-scid (Taconic) mice as previously described [29]. Tumors were harvested at autopsy for Western blot analysis. Sections of paraffin-embedded tumors on slides were processed for immunohistochemistry as previously described [30].

### Statistical analysis

Statistical analyses were performed with Student’s *t* test and ANOVA models using Systat 13 (Systat Software, Chicago, IL). *P* values of less then 0.05 were considered significant.

## Results

### Identification of a potent mTORC2-specific inhibitor

To identify small molecules which specifically target mTORC2 we sought to disrupt the Rictor-mTOR interaction. Rictor is an obligate regulatory subunit of mTORC2 [31], and inhibition of Rictor expression has been demonstrated to block mTORC2 assembly and activity [32]. Towards this end, we utilized an approach developed by Golemis and Tamanoi [33, 34], and engineered a yeast-two hybrid screen utilizing a drug hyperpermeable strain (S1 Fig), to identify inhibitors of the Rictor-mTOR protein-protein interaction. Yeast dependent on the interaction of the full-length human mTOR and Rictor proteins for growth on selective media were screened against the NCI/DTP small molecule compound library (>145,000 diversity-oriented compounds) (Fig 1A). As shown in Fig 1B, we identified compounds which inhibited growth under these conditions and as a counterscreen, we ruled out potential inhibitors that also blocked the interaction of SV40 large T-antigen and p53 [35]. These compounds were considered non-specific and generally toxic to yeast and were omitted from further study. From this screen we identified several compounds which blocked Rictor-mTOR association in yeast (Fig 1C). Additionally, some of these compounds were predicted to be toxic in mammalian cells and were not pursued. CID613034 was chosen for further study, as it displayed minimal cytotoxicity to normal human neurons (S2 Fig). We subsequently determined the effects of this compound in GBM cell lines, in terms of its ability to specifically block mTORC2 formation and activity. As shown in Fig 1D, CID613034, in a concentration-dependent manner, inhibited mTORC2 *in vitro* kinase activity. CID613034 also blocked the association of Rictor with mTOR in immunoprecipitates of mTOR from U87 cells treated with the inhibitor (Fig 1E). The ability of the compound to block Rictor-mTOR association was specific as Raptor-mTOR binding was unaffected. In U87 and LN229 GBM lines, CID613034 markedly inhibited phosphorylation of known mTORC2 substrates such as phospho-S^473^-AKT, phospho-T^346^-NDRG1 and phospho-S^657^-PKCα, while having no discernible effect on the levels of phospho-T^389^-S6K, a mTORC1 specific phospho-site. Moreover, in time-course and dose-response experiments (S3 Fig), CID613034 inhibited mTORC2 signaling in a concentration-dependent manner with marked inhibition of activity within 2 hours of treatment in GBM cells, while having no significant effects on mTORC1 activity. These data suggest that CID613034 is a potent mTORC2-specific inhibitor.

**Fig 1:** Identification of compounds which inhibit mTORC2 activity in glioblastoma cells. **(**A) Yeast two-hybrid assay configuration used to screen for inhibitors of the human Rictor-mTOR interaction. Full-length human Rictor fused to the Gal4-DNA-binding domain and mTOR fused to the Gal4-activation domain was expressed in yeast containing reporters harboring *Gal4* upstream activating sequences (UAS). (B) Screening of compounds which block Rictor/mTOR association. Yeast expressing either p53-DBD and SV40 large T antigen-AD fusions or Rictor-DBD and mTOR-AD fusions were plated. Compounds were pinned onto the plate surfaces and examined for halo formation (red circles). Compounds which inhibited Rictor/mTOR-mediated growth on selective media while having little or no effects on p53/T antigen-mediated growth were considered specific. Compounds which blocked growth of both strains were considered nonspecific and exhibited general antifungal activity. **(**C) Structures of compounds which inhibit Rictor/mTOR association. **(**D) CID613034 inhibits mTORC2 *in vitro* kinase activity. mTORC2 kinase reactions were performed using GST-tagged AKT as a substrate with the indicated concentrations of inhibitor. Reactions were subsequently immunoblotted for phospho-S^473^-AKT and GST-tagged AKT. **(**E) CID613034 blocks binding of Rictor to mTOR in LN229 cells. Cells were treated with 5 mM Antimycin (control compound), 50 nM CID613034 or 20 nM rapamycin for 15 min and mTOR immunoprecipitated. Immunoprecipitations were then immunoblotted for the indicated proteins. **(**F) mTORC2 signaling is inhibited in GBM lines following 24 h exposure to CID613034. LN229 or U87 cells were treated with 100 nM of inhibitor as shown and lysates immunoblotted for the indicated proteins. Data shown are representative of experiments repeated two times.

### Anti-GBM effects of CID613034 *in vitro*

To determine the response of GBM cell lines to CID613034, we performed XTT assays in U87 and LN229 cells at various concentrations of inhibitor over the course of 96 hours. As shown in Fig 2A, CID613034 treatment resulted in dose-dependent cytotoxicity in both lines. Treatment with the compound also had marked effects on GBM motility and invasive characteristics consistent with the blockade of mTORC2 activity, which is known to regulate these properties [14]. To initially determine whether CID613034 affected the ability of GBM cells to form colonies in soft agar, we treated U87 and LN229 cells with the inhibitor in clonogenic growth assays. As shown in Fig 2B, clonogenic growth of both U87 and LN229 were markedly inhibited by the compound. To determine if CID613034 treatment affected cell migration, we assessed the ability of CID613034 treated cells to traverse a vitronectin-coated or fibronectin-coated Boyden chamber as compared to chambers coated with BSA as a control. In a dose-dependent fashion CID613034 significantly inhibited the numbers of cells that migrated towards vitronectin or fibronectin-coated surfaces as compared to control BSA-coated surfaces (Fig 2C). We also tested whether CID613034 affected the ability of U87 or LN229 cells to invade Matrigel. As shown in Fig 2D, the compound significantly blocked migratory ability with increasing concentration. Finally, we examined the cell-cycle phase distributions of U87 and LN229 cells treated with the inhibitor. As shown in Fig 2E, CID613034 increased the percentage of cells in G_1_/G_0_ with a concomitant reduction in S-phase and unchanged G_2_/M numbers. CID613034 treatment also induced significant apoptosis in these cells relative to untreated controls (Fig 2F). Taken together, these data demonstrate significant inhibitory effects of CID613034 on GBM cell growth, migration and invasive properties.

**Fig 2:** Anti-GBM effects of CID613034 in cell lines. **(**A) Inhibition of GBM cell line proliferation following culture with CID613034 (black, 0 μM; blue, 0.5 μM; red, 1 μM; green, 2 μM) for the indicated time points. (*, *P*< 0.05). Data represent mean ±S.D. of three independent experiments. (B) CID613034 exposure inhibits anchorage-independent growth. Cells were suspended in soft agar to evaluate anchorage independent growth in the presence of the indicated concentrations of inhibitor and colonies counted after 14 days of growth. Data represent mean +S.D. of three independent experiments. (C) Migration of U87 and LN229 cells in the presence of the indicated concentration of CID613034. Cells were seeded into Boyden chambers and allowed to migrate towards BSA (white bars), vitronectin (grey bars) or fibronectin (black bars) (*, *P*<0.05). Data represent mean +S.D. of three independent experiments. (D) Invasive potential of U87 or LN229 cells in the presence of the indicated concentrations of CID613034 migrating through matrigel. Data represent mean +S.D. of three independent experiments. (E) Cell-cycle phase distributions were determined on the indicated lines treated with CID613034 as shown. One of three experiments with similar results is shown. (F) Percent apoptotic cells as determined via annexin V-FITC staining. Data represent mean +S.D. of three independent experiments.

### Sensitivity to CID613034 is dependent on relative Rictor or mSIN1 levels in GBM

The relative expression of Rictor has been demonstrated to regulate the formation of mTORC2 and its activity [13, 14]. To determine whether Rictor expression can alter the sensitivity of GBM cells to CID613034 we initially determined Rictor levels in several cell lines and attempted to correlate relative expression with drug sensitivity. As shown in Fig 3A, Rictor expression was varied in these lines and expression levels were quantified via densitometry and normalized to levels observed in U87 cells. In Fig 3B, the relative Rictor expression in the lines tested was high in most cases except for H4, U373 and U138 which displayed low Rictor levels and LN229 and M059J in which expression was at intermediate levels. We subsequently tested these cell lines in XTT assays to determine the cellular responses to CID613034 over a wide range of concentrations (Fig 3C). A significant inverse correlation was observed between the IC_50_ for CID613034 and relative Rictor expression in the cell lines tested (Fig 3D) demonstrating that lines which harbored elevated levels of Rictor were the most sensitive to the drug, while those with low Rictor expression were relatively resistant. We also tested the effects of CID613034 on U87 cells in which Rictor was knocked-down via stable overexpression of an shRNA targeting Rictor or cells that stably overexpressed Rictor via an expression construct (Fig 3E). U87 cells stably overexpressing Rictor were very sensitive to CID613034 while U87_shRictor_ cells were markedly resistant. Similarly, we tested the sensitivity of wt and mSIN1-null MEFs to CID613034 and these cells also displayed differential sensitivities to the compound, as wt MEFs were significantly more sensitive as compared to mSIN-null MEFs at concentrations over 0.25 μM (Fig 3F).

**Fig 3:** Sensitivity to CID613034 is dependent on Rictor or SIN1 expression. **(**A) Steady-state Rictor expression levels in GBM lines. Lysates from the indicated lines were immunoblotted for Rictor and actin levels. (B) Quantification of Rictor expression levels from (A) as determined by densitometric analyses. Relative Rictor expression in U87 cells was arbitrarily assigned a value of 1. Rictor expression in all cell lines is shown as mean +S.D., n = 3. (C) XTT proliferation assays performed on eleven GBM lines with increasing concentration of CID613034 at 72 h. (D) Correlation between CID613034 sensitivity and IC_50_ determined for all GBM cell lines treated with CID613034 for 72 h and shown as means of 3–5 individual experiments. Relative Rictor expression was obtained from (B) above. (E) Sensitivity of U87, U87shRictor and U87-Rictor GBM cells to CID613034 treated with the indicated concentrations at 72 h. Data represent mean ±S.D. of three independent experiments. *, *P* < 0.05 (F) Sensitivity of wt SIN1 and SIN1-null MEFs to increasing concentrations of CID613034 at 48 h. Data represent mean ±S.D. of three independent experiments. *, *P* < 0.05

### SAR studies derive active analogs of CID613034

A series of thirty analogs were synthesized based on the structure of CID613034 (also designated JR-AB2-000) to explore the SAR properties of the inhibitor. Modifications were made to all functional groups of the molecule as shown in Fig 4 (see also S4 Fig), and we determined whether these analogs effected mTORC2 signaling and anti-GBM responses. These data are summarized in Table 1. In Fig 4, showing analogs with modifications to the left-side of the molecule (**R**_**1**_), no significant improvements in mTORC2 signaling blockade, as determined by the degree of p-S^473^-AKT inhibition relative to values obtained with the parent inhibitor, were observed. Additionally, no alterations in IC_50_ or apoptosis values were observed with these analogs suggesting that this region of the molecule was not critical for inhibition of mTORC2. Within the analogs containing modifications to the right-side of the molecule (**R**_**2**_), JR-AB2-005 displayed a significant increase in IC_50_; however p-S-^473^-AKT levels and the degree of apoptosis in cells following exposure were unaffected. The analog JR-AB2-011 however, markedly reduced mTORC2 signaling (see also S5 Fig) and IC_50_ while enhancing apoptotic levels in GBM cells compared to the parent compound. Similarly, analog JR-AB2-030 also blocked mTORC2 signaling and lowered the IC_50_ value while increasing apoptosis levels, albeit to a lesser degree then analog JR-AB2-011. Additional analogs were synthesized shown in Fig 4 (**R**_**3**_ modifications and analogs JR-AB2-027 thru -029); however none of these significantly improved mTORC2 signal blockade or anti-GBM properties as compared to the parent inhibitor. Moreover, we determined the *in vitro* cytotoxicities of analogs JR-AB2-011 and JR-AB2-030 relative to JR-AB2-000 in human neurons (not shown). JR-AB2-011 displayed the least toxicity to normal neurons with no significant cytotoxic effects for concentrations up to 10 mM and was chosen for further study.

**Fig 4:** Synthesis of JR-AB2-000 (CID613034) analogs. Thirty analogs were synthesized with the indicated group modification shown and further detailed in Table 1. Analog identification numbers are shown below the structures corresponding to analogs where a particular functional group is modified. Detailed synthetic procedures and NMR spectra are described in supplementary Materials and methods.

**Table 1:** Summary of anti-GBM effects of CID613034 analogs.

Compound	Chemical formula	^§^ mTORC2 activity (fold decrease)	IC_50_ (μM)	% Apoptosis (1 μM)
**JR-AB2-000**	**C**_**19**_**H**_**19**_**Cl**_**2**_**N**_**3**_**OS**	**1.0**	**1.76±0.51**	**18.2**
**JR-AB2-001**	**C**_**18**_**H**_**17**_**Cl**_**2**_**N**_**3**_**OS**	**0.95**	**1.30±0.11**	**19.4**
**JR-AB2-002**	**C**_**20**_**H**_**21**_**Cl**_**2**_**N**_**3**_**OS**	**1.10**	**1.62±0.37**	**12.6**
**JR-AB2-003**	**C**_**20**_**H**_**24**_**N**_**4**_**O**_**2**_**S**	**0.94**	**2.46±0.49**	**15.7**
**JR-AB2-004**	**C**_**19**_**H**_**19**_**Cl**_**2**_**N**_**3**_**S**_**2**_	**1.05**	**1.51±0.82**	**11.0**
**JR-AB2-005**	**C**_**18**_**H**_**17**_**Cl**_**2**_**N**_**3**_**O**_**2**_**S**	**1.19**	**5.77±0.63**	**13.8**
**JR-AB2-006**	**C**_**19**_**H**_**19**_**Cl**_**2**_**N**_**3**_**O**_**2**_	**1.05**	**1.05±0.36**	**11.5**
**JR-AB2-007**	**C**_**17**_**H**_**15**_**Cl**_**2**_**N**_**3**_**OS**	**1.10**	**1.48±0.95**	**10.2**
**JR-AB2-008**	**C**_**19**_**H**_**20**_**Cl**_**2**_**N**_**4**_**OS**	**1.36**	**1.86±0.21**	**12.7**
**JR-AB2-009**	**C**_**18**_**H**_**17**_**Cl**_**2**_**N**_**3**_**OS**	**1.05**	**1.93±0.54**	**13.9**
**JR-AB2-010**	**C**_**18**_**H**_**17**_**Cl**_**2**_**N**_**3**_**OS**	**1.17**	**1.37±0.68**	**17.4**
**JR-AB2-011**	**C**_**17**_**H**_**14**_**Cl**_**2**_**FN**_**3**_**OS**	**3.94**	**0.31±0.17**	**36.3**
**JR-AB2-012**	**C**_**13**_**H**_**15**_**Cl**_**2**_**N**_**3**_**OS**	**1.18**	**0.96±0.14**	**16.4**
**JR-AB2-013**	**C**_**18**_**H**_**15**_**Cl**_**2**_**N**_**3**_**OS**	**1.12**	**2.15±0.10**	**20.2**
**JR-AB2-014**	**C**_**22**_**H**_**17**_**Cl**_**2**_**N**_**3**_**OS**	**1.24**	**1.39±0.37**	**19.7**
**JR-AB2-015**	**C**_**20**_**H**_**21**_**Cl**_**2**_**N**_**3**_**OS**	**1.03**	**1.19±0.63**	**10.6**
**JR-AB2-016**	**C**_**20**_**H**_**17**_**Cl**_**2**_**N**_**3**_**O**	**1.29**	**1.50±0.24**	**11.5**
**JR-AB2-017**	**C**_**21**_**H**_**18**_**Cl**_**2**_**N**_**2**_**O**	**1.05**	**1.72±0.93**	**16.1**
**JR-AB2-018**	**C**_**19**_**H**_**21**_**N**_**3**_**OS**	**1.67**	**1.14±0.59**	**12.2**
**JR-AB2-019**	**C**_**19**_**H**_**20**_**ClN**_**3**_**OS**	**1.93**	**1.28±0.83**	**15.7**
**JR-AB2-020**	**C**_**19**_**H**_**20**_**ClN**_**3**_**OS**	**1.58**	**2.11±0.38**	**17.8**
**JR-AB2-021**	**C**_**19**_**H**_**20**_**FN**_**3**_**OS**	**1.59**	**1.83±0.15**	**10.2**
**JR-AB2-022**	**C**_**20**_**H**_**23**_**N**_**3**_**OS**	**1.13**	**1.42±0.32**	**15.9**
**JR-AB2-023**	**C20H23N3O2S**	**1.24**	**0.98±0.24**	**16.3**
**JR-AB2-024**	**C23H23N3OS**	**1.65**	**1.26±0.27**	**26.0**
**JR-AB2-025**	**C15H21N3OS**	**1.37**	**1.39±0.48**	**17.5**
**JR-AB2-026**	**C17H25N3OS**	**1.18**	**2.82±0.75**	**11.3**
**JR-AB2-027**	**C20H20Cl2N2OS**	**1.41**	**1.86±0.39**	**12.2**
**JR-AB2-028**	**C19H18Cl2N2O2S**	**1.30**	**2.10±0.29**	**14.6**
**JR-AB2-029**	**C20H21Cl2N3OS**	**1.72**	**1.14±0.38**	**11.7**
**JR-AB2-030**	**C17H14BrCl2N3OS**	**2.69**	**0.57±0.20**	**20.5**

§, Fold decrease mTORC2 activity as determined by densitometric quantification of immunoblots probed for phospho-S^473^-AKT abundance in LN229 cells treated with 1 μM analog for 24 h as compared to values obtained with parent compound (JR-AB2-000) under identical conditions. No significant alterations in p-T^389^-S6K levels were observed for any of the analogs (1 μM, 24 h) as compared to untreated controls (not shown). For each analog the IC_50_ was determined via XTT proliferation assays as in Fig 3C and 3D. Data represent mean ±S.D. of three independent experiments. Percent apoptosis was determined for LN229 cells treated with analog (1μM) at 48 h via annexin V-FITC staining. One of three experiments with similar results is shown.

### JR-AB2-000 or analog JR-AB2-011 inhibit association of Rictor to mTOR

To begin to investigate the mechanism of action of JR-AB2-000 and its analog JR-AB2-011 we performed SPR analyses of JR-AB2-000 binding to either immobilized Rictor, mTOR or mSIN1. As shown in Fig 5A (left-panel), JR-AB2-000 selectively bound to Rictor and reached equilibrium rapidly. The K_d_ was determined from steady-state binding associations and was calculated at 1 μM. Contrastingly, JR-AB2-000 was unable to bind mTOR or mSIN1, another regulatory subunit of mTORC2. We were unable to observe mTOR binding to immobilized Rictor, however in the reverse configuration immobilized mTOR bound Rictor with a calculated K_d_ of 257 nM (Fig 5A, right panel). In competitive SPR assays in which immobilized mTOR was allowed to bind analyte containing preincubated Rictor bound to either JR-AB2-000 or JR-AB2-011, the latter inhibitor showed increased potency and a 6–7 fold improved binding affinity to Rictor (JR-AB2-011; IC_50_ = 0.36 μmol/L; K_i_ = 0.19 μmol/L) in comparison with the parent compound (JR-AB2-000; IC_50_ = 1.64 μmol/L; K_i_ = 1.46 μmol/L) (Fig 5B, left panel). To further confirm specificity, we preincubated each of the inhibitors with either Raptor (mTORC1 subunit), mLST8 or Deptor (both mTORC1 & 2 subunits) and these reaction mixtures were passed over immobilized mTOR. Neither JR-AB2-011 or JR-AB2-000 significantly effected the binding of Raptor, mLST8 or Deptor to immobilized mTOR (Fig 5B, middle & right panels). Additionally, we determined the ability of JR-AB2-011 or JR-AB2-000 to inhibit mTOR-Rictor association in a pull-down assay utilizing Flag-mTOR and myc-Rictor. As shown in Fig 5C, both inhibitors blocked the ability of bead bound Flag-mTOR to bind myc-Rictor. JR-AB2-011 appeared to more effectively block mTOR-Rictor association at the highest concentration of inhibitor relative to the parent compound in this assay. Taken together, these results support the notion that the analog JR-AB2-011 and its parent bind Rictor and specifically block mTOR association. Additionally, these data suggest that JR-AB2-011 more effectively inhibits mTOR binding relative to the parent compound.

**Fig 5:** JR-AB-000 and JR-AB-011 bind to Rictor and prevent Rictor-mTOR association. **(**A) Surface plasmon resonance analysis of JR-AB-000 binding to immobilized Rictor, mSIN1 or mTOR as indicated (left panel). Binding sensorgrams of immobilized mTOR with Rictor over the indicated concentration range (right panel). The K_on_, K_off_ and K_d_ were calculated by simultaneous non-linear regression using a 1:1 binding model and BIAevaluation 3.1 software. (B) Competitive binding curves of Rictor-mTOR association in the absence or presence of JR-AB2-011 or JR-AB2-000 as indicated (left panel). Analysis of selectivity of JR-AB2-011 (middle panel) or JR-AB2-000 (right panel) binding to Rictor, Raptor, mLST8 or Deptor as shown. Samples were preincubated with inhibitors and Rictor, Raptor, mLST8 or Deptor proteins as indicated and run over sensor chip containing immobilized mTOR. The IC_50_ values were calculated using the response units at the dissociation phase. (C) mTOR-Flag coupled beads binding to myc-Rictor in the presence of increasing JR-AB2-011 (top panels) or JR-AB2-000 (bottom panels). myc-Rictor was incubated with inhibitor for 1 h followed by incubation with FLAG agarose beads coupled to mTOR-Flag (mTOR-Flag beads). Binding of myc-Rictor to mTOR-Flag beads (Rictor-mTOR-Flag beads) was detected by immunoblotting with an anti-myc mAb. The amount of protein bound to FLAG agarose beads was detected with an anti-Flag mAb (loading control). Immunoblots were quantified via densitometric analyses and graphs are shown to the right of the blots. Three independent experiments were performed and one representative result is shown.

### Effects of JR-AB2-011 therapy in GBM xenografts

To determine the *in vivo* effects of JR-AB2-011, we conducted xenograft studies utilizing LN229 cells in mice. Mice were subcutaneously implanted with tumor cells and when tumors were palpable (~200 mm^3^), mice were randomized into treatment groups receiving vehicle, JR-AB2-011 (4 mg/kg/d) and JR-AB2-011 (20 mg/kg/d). As shown in Fig 6A, mice receiving JR-AB2-011 at either dosing regimen displayed marked inhibition of tumor growth rate (JR-AB2-011 at 4 mg/kg/d; 74% inhibition at end of dosing period; tumor growth delay 10.0 days; JR-AB2-011 at 20 mg/kg/d; 80% inhibition at end of dosing period; tumor growth delay 12.0 days) as compared to mice receiving vehicle alone. Consistent with the effects on xenograft growth, overall survival of mice at either JR-AB2-011 dosing regimen was significantly extended relative to vehicle treated mice. Notably, mice tolerated both of these dosing regimens without obvious short or long-term toxicity or weight loss. Blood cell counts were not affected by JR-AB2-011 (S6 Fig). A significant reduction in tumor proliferation (Ki-67 staining of harvested tumors) was observed at both dosing regimens (Fig 6C, upper left panel). The induction of apoptotic cell death was monitored by TUNEL staining and JR-AB2-011 at both dosing regimens markedly enhanced apoptosis, supporting the increases in apoptotic death observed *in vitro* with the parent compound (Fig 6C, upper right panel; see also Fig 2F). The ratio of phospho-S^473^-AKT to total AKT was significantly reduced in tumors at both doses of JR-AB2-011, while the ratio of phospho-T^389^-S6K to total S6K was not significantly altered (Fig 6C, lower left and right panels).

**Fig 6:** Effects of JR-AB2-011 treatment on GBM tumor growth in mice. **(**A) Tumor burden of SCID mice implanted with LN229 cells and treated with the indicated schedules of vehicle, JR-AB2-011 (4 mg/kg/d) and JR-AB2-011 (20 mg/kg/d) for ten consecutive days and tumor growth assessed every two days following initiation of treatment (start, day 0). *, *P* < 0.05, significantly different from vehicle, JR-AB2-011 (4 mg/kg/d) and JR-AB2-011 (20 mg/kg/d). (B) Overall survival of subcutaneous LN229 tumors receiving the indicated treatment schedules. (C) Ki-67 positive cells were identified via immunohistochemical staining of sections prepared from harvested tumors at day 12 following initiation of treatment regimens (upper left panel). Apoptotic cells were identified by TUNEL assays of sections prepared from harvested tumors at day 12 following initiation of treatment regimens (upper right panel). Data are expressed as the number of positive apoptotic bodies divided by high power field (hpf; 10–12 hpf/tumor). Values are means +S.D., *, *P* < 0.05. Phospho-S^473^-AKT/total AKT protein ratio levels in tumors (lower left panel). Values are means ±S.D., *, *P* < 0.05, significantly different from vehicle, JR-AB2-011 (4 mg/kg/d) and JR-AB2-011 (20 mg/kg/d). Phospho-T^389^-S6K/total S6K protein ratio levels in tumors (lower right panel). Values are means ±S.D., *, *P* < 0.05, significantly different from vehicle, JR-AB2-011 (4 mg/kg/d) and JR-AB2-011 (20 mg/kg/d). Protein levels were quantified by Western analyses of harvested tumors from mice with the corresponding treatments as indicated and described in Material and methods.

## Discussion

There is increasing evidence to support dysregulation of mTORC2/AKT signaling in the pathogenesis and progression of several cancers [8, 36]. Thus, activation of mTORC2, downstream of PI-3K or Rac1, or as a result of Rictor amplification or alterations in protein stability may serve as a nodal point in cell signaling highlighting its potential as a drug target. In this report, we describe the identification and action of an inhibitor of mTORC2 and demonstrate its significant anti-GBM activity. SAR studies identified an improved inhibitor which also demonstrated significant anti-GBM properties *in vitro* and *in vivo*. Experiments addressing the mechanism of action of the inhibitors demonstrate that the inhibitors bind Rictor in such a manner as to preclude subsequent mTOR association. Our studies are most consistent with the hypothesis that these inhibitors likely disrupt Rictor-mTOR binding by binding to Rictor at a site(s) either directly involved in mTOR binding or at a site which allosterically prevents mTOR association. The improved ability of the SAR optimized analog JR-AB2-011 to block mTORC2 signaling may be due to the greater apparent affinity of JR-AB2-011 for Rictor. This is supported by SPR experiments in Fig 5B (left panel), in which the K_i_ for JR-AB2-011 was found to be 6–7 fold lower relative to JR-AB2-000 in competitive binding assays.

Mammalian TORC2 is ~1.3 MDa and contains two copies of each of six subunits: mTOR, mLST8, Rictor, mSIN1, Deptor and PRR5 or its paralog PRR5L [37]. Besides mTOR, Rictor is the largest subunit of TORC2. Disruption or RNAi-mediated depletion of Rictor results in the disassembly of TORC2 suggesting that Rictor performs a critical scaffolding function [38]. In our binding studies both the parent and JR-AB2-011 inhibitors bound to Rictor and prevented the association of mTOR, consistent with the notion that these compounds are able to inhibit assembly of mTORC2. It is unknown if JR-AB2-011 can also result in the disassembly of preformed mTORC2. While unlikely, we also cannot rule out additional possible effects of JR-AB2-011 on PRR5 function such that mTORC2 activity is impaired. Future mechanistic studies will be required to address these questions.

There are currently three classes of compounds which can inhibit mTORC2 activity (ATP-competitive, dual PI-3K/mTOR inhibitors and rapamycin); however none of these inhibitors are specific. All suffer from the potential limitation of blocking mTORC1 and inactivating negative feedback loops resulting in the activation of AKT, even in the context of mTORC2 inhibition [9]. The inhibitors described here are specific for mTORC2 in that mTORC1 was apparently unaffected by exposure, as we monitored one of the most well established markers of mTORC1 activity, phospho-T^389^-S6K, as a readout. Additionally, we noted that phospho-S^312^ and total IRS1 levels were unchanged suggesting that at least the S6K/IRS1/PI-3K feedback loop remained intact in the presence of CID613034 (S3A Fig). MAPK activation is also downstream of this feedback loop and ERK activity was unresponsive to CID613034 (S3B Fig).

Our data demonstrated that an important determinant of sensitivity to CID613034 is relative Rictor or SIN1 expression. This is most likely a result of increased mTORC2 formation, as increased expression of these subunits would be expected to promote the nucleation of signaling competent mTORC2 kinases. Since our data demonstrated that these inhibitors bind Rictor, it is possible that post-translational modifications of Rictor, such as phosphorylation or acetylation may additionally be critical determinants of sensitivity for these compounds. Indeed, recent experiments show that glucose-dependent acetylation of Rictor promotes resistance to EGFR, PI-3K or AKT targeted therapies in GBM [39]. It is conceivable that such modifications to Rictor may affect the affinity of JR-AB2-011 for its putative binding site. Another important consideration is the possibility that CID613034 or JR-AB2-011-bound Rictor may exert effects on several mTORC2-independent signaling cascades regulating cell proliferation and motility [15, 40–42]. Future studies with these compounds examining the mTORC2-independent functions of Rictor will be necessary.

Recent studies have described the development of strategies to specifically inhibit TORC2 acutely in yeast utilizing reverse chemical genetics [37]. To investigate the selective pharmacology of TORC2 blockade, Kliegman *et al*., engineered an allele of TOR2 which accepted an orthogonal kinase inhibitor that did not inhibit TOR1 [43]. These studies implicated known regulatory relationships between TORC2 and sphingolipid biosynthesis and also identified novel regulation of the pentose phosphate pathway by TORC2. Rispal *et al*., characterized the downstream effectors of TORC2 by engineering TORC1 to be resistant to the ATP-competitive TOR inhibitor NVP-BHS345 and subsequent treatment with the compound specifically blocked TORC2 [44]. Phosphoproteomic analyses elucidated regulatory effects of TORC2 on actin polarization and endocytosis, via the phospholipid flippase kinases Fpk1 and Fpk2 and identified a broad spectrum of potential TORC2 effectors. We envision the combined use of JR-AB2-011 and phosphoproteomics in mammalian cells may permit a similarly comprehensive analysis of mTORC2 substrates.

In summary, we have identified inhibitors of mTORC2 activity which target the regulatory subunit Rictor. We have demonstrated that these inhibitors have broad anti-GBM effects *in vitro* and in xenograft experiments. SPR and mTOR-bead pull-down experiments suggest that CID613034 and JR-AB2-011 specifically bind to Rictor and block association with mTOR. These results demonstrate that mTORC2 is a compelling target in GBM and support the use of these compounds in further dissection of mTORC2-mediated signaling processes.

## Supporting information

S1 Fig (A) Schematic diagram of kanMX PCR disruption cassettes used to knockout the *pdr1*and *pdr3* loci via homologous recombination. Following transformation, the presence of the cassette was confirmed via amplification using a gene-specific primer and a primer within the kanMX ORF (primer arrows shown on schematic and arrow next to gel shows appropriate sized PCR products amplified from the indicated transformant). Subsequently, the Cre recombinase was expressed to remove the kanMX cassette. **(**B) Following knockout of the *Pdr* genes, HA-tagged versions of Hxt9p and Hxt11p under control of the *Cup1* promoter were stably integrated and induced by the presence of copper in the media. (C) Drug sensitivities of the parental and modified drug sensitive yeast two-hybrid strain on solid (above) or liquid (below) media in the presence of the indicated inhibitor and copper to induce the Hxt transporters. Open circles denote values for the parental strain, while closed circles denote growth in the presence of the indicated inhibitor.
(TIFF)

S2 Fig TUNEL staining of human neurons treated with increasing concentrations of CID613034 (left panel) or JR-AB2-011 (right panel) following 48 h exposure. Data shown are mean +S.D., n = 3.
(TIF)

S3 Fig Kinetics and dose-response of CID613034 mediated-inhibition of mTORC2 signaling in LN229 cells. (A) LN229 cells were treated with CID613034 (1 μM) for the indicated time points and lysates immunoblotted for the indicated proteins. (B) LN229 cells were treated with CID613034 at the indicated concentrations for 2.5 h and protein lysates immunoblotted for the indicated proteins.
(TIF)

S4 Fig Chemical structures of CID613034 analog modifications. (TIF)

S5 Fig Treatment of U87 and LN229 GBM cells with JR-AB2-011 (1 μM) for 24 h and lysates immunoblotted for the indicated proteins. (TIF)

S6 Fig Peripheral blood RBC and WBC counts in mice (5 mice/group) treated with daily IP injections (10 days) of 0, 4 or 20 mg/kg/d of JR-AB2-011. Data are expressed as percent of control mice that received vehicle only and assigned 100%.
(TIF)

S1 File Supplemental materials and methods. (PDF)
